# Identification of Differentially Expressed Genes Reveals BGN Predicting Overall Survival and Tumor Immune Infiltration of Gastric Cancer

**DOI:** 10.1155/2021/5494840

**Published:** 2021-11-26

**Authors:** Weizhi Chen, Zhongheng Yang

**Affiliations:** ^1^Department of Radiology, The First Affiliated Hospital of Jinzhou Medical University, 121001, China; ^2^Department of Stomatology, The First Affiliated Hospital of Jinzhou Medical University, 121001, China

## Abstract

Gastric cancer (GC) is one of the most widely occurring malignancies worldwide. Although the diagnosis and treatment strategies of GC have been greatly improved in the past few decades, the morbidity and lethality rates of GC are still rising due to lacking early diagnosis strategies and powerful treatments. In this study, a total of 37 differentially expressed genes were identified in GC by analyzing TCGA, GSE118897, GSE19826, and GSE54129. Using the PPI database, we identified 17 hub genes in GC. By analyzing the expression of hub genes and OS, MFAP2, BGN, and TREM1 were related to the prognosis of GC. In addition, our results showed that higher levels of BGN exhibited a significant correlation with shorter OS time in GC. Nomogram analysis showed that the dysregulation of BGN could predict the prognosis of GC. Moreover, we revealed that BGN had a markedly negative correlation with B cells but had positive correlations with CD8^+^ T cells, CD4^+^ T cells, macrophages, neutrophils, and dendritic cells in GC samples. The pan-cancer analysis demonstrated that BGN was differentially expressed and related to tumor-infiltrating immune cells across human cancers. This study for the first time comprehensively revealed that BGN was a potential biomarker for the prediction of GC prognosis and tumor immune infiltration.

## 1. Introduction

Gastric cancer (GC) ranks fifth amid the widely occurring malignancies worldwide and is the third primary inducer of carcinoma-related mortality [1]. GC belongs to a disease involving environmental and genetic factors, which both exert an effect on GC occurrence and development [1, 2]. High intake of traditional salt-preserved foods and salt and low intake of fresh fruits and vegetables are likely to be related to tumorigenesis of GC [1–3]. Smoking is also one external risk factor easily contributing to GC. Additionally, Helicobacter pylori (*H*. *pylori*) and Epstein-Barr virus (EBV) are the main risk factors for GC development [1, 2]. Nevertheless, the distribution of histological subtypes of GC and the frequencies of *H*. *pylori*- and EBV-related GC vary worldwide [4–6]. The genetic diffuse GC accounts for approximately 1-3% of GC cases [7]. Host factors such as cytokine gene polymorphisms and bacterial factors are related to the increase in inflammation intensity and progression risk [8, 9]. Present GC treatments are composed of surgery [10], radiotherapy [11], neoadjuvant chemotherapy [12], and immunotherapy [13]. Early GC patients' survival rate attains 90%. Detection and diagnosis of GC at the early stage, however, is not easy, leading to an obvious decline in the survival rate after diagnosis [14]. Herein, it is of great significance to uncover potential biomarkers for GC diagnosis and prognosis and to explore treatment targets for early GC.

BGN is an essential constituent of the extracellular matrix (ECM) that exhibited an association with several human carcinomas [15], including GC [16], esophageal squamous cell carcinoma [17], pancreatic carcinoma [18], colon carcinoma [19], and neoplasms in blood vessels. In terms of mechanism, it has been proved that proteoglycans could facilitate cell proliferation, affect migration, and weaken cell adhesion via interacting with proteins in the intracellular matrix and extracellular matrix. Hu et al. [16] found that BGN was greatly upregulated in the tissues of GC compared to the adjacent nontumor gastric tissues and was related to the metastasis of axillary lymph nodes, the depth of tumor invasion, and the metastasis (TNM) stage of tumor nodes. What is more, BGN boosted the invasion ability of GC cells via motivating the FAK signaling pathway. Subsequently, it was suggested that the mechanism of BGN-induced GC angiogenesis was that BGN interacted with TLR2/4 via the NF-*κ*B-dependent activation to promote the formation, migration, and proliferation of endothelial cell tubes [15]. However, the expression pattern and potential roles of BGN in GC remained to be unknown.

Recently, some studies have implied that integrating several biomarkers into a single model presented a relatively higher prediction accuracy in comparison with a single biomarker [19]. In our study, we extracted RNA-Seq data from TCGA and multiple microarray-based datasets to identify the differentially expressed genes (DEGs) between GC tissues and adjacent nontumor tissues. By using multiple bioinformatics methods, we identified that BGN was a potential biomarker for GC.

## 2. Materials and Methods

### 2.1. Microarray Data Information

The gene expression data, clinicopathological characteristics, and prognosis information of GC patients were obtained from TCGA database. We extracted clinicopathological characteristics from 358 GC cases and 51 adjacent normal samples. Ten GC and 10 normal samples were contained in the GSE118897 [20] dataset, 12 GC and 15 normal samples were included in the GSE19826 [21] dataset, and 111 GC and 23 normal samples were involved in the GSE54129 dataset.

### 2.2. DEG Identification

Software R (version 3.6.3, https://www.r-project.org) and “*limma*” packages (http://www.bioconductor.org/) were applied to select the DEGs, with adjusted *p* value < 0.05 and ∣log2 fold change (FC) | ≥2. The DEGs with *p* < 0.1 and FC > 1.5 (∣log2FC | >0.585) were considered to be differentially expressed [22].

### 2.3. GO and KEGG Pathway Enrichment Analyses

Gene Ontology (GO) and KEGG pathway enrichment analyses were utilized to evaluate molecular interaction and relation pathways by DAVID (https://david.ncifcrf.gov/home.jsp) and GSEA software (version 3.0). *p* < 0.05 and gene counts ≥ 5were thought to be the cutoff criteria.

### 2.4. Protein-Protein Interaction (PPI) Network Construction

The PPI network was established by the STRING database. Significant interaction meant the combined score > 0.4.

### 2.5. Establishing and Validating the Nomogram

In order to predict STAD patients' clinical outcomes, we made use of the R package “rms” to establish a nomogram consisting of clinical factors and risk signatures. In addition, the performance and prediction accuracy of the nomogram was measured to plot calibration curves.

For the establishment of the nomogram, we carried out univariate and multivariate Cox regression analyses to determine the proper terms. The forest displayed the *p* value, HR, and 95% CI of individual variables by the “forestplot” R package. In light of the data of multivariate Cox proportional hazards analysis, we generated a nomogram to forecast the *X*-year overall recurrence rate. The nomogram offered a graphical representation regarding these factors, which could be utilized to reckon the recurrence risk for individual patients by means of each risk factor-associated point.

### 2.6. Survival Analysis

The survival and survminer packages in R were employed to compare the OS between groups by Kaplan-Meier analysis. The risk model's accuracy that was used for predicting the OS of patients was exploited to form a ROC curve via the survival ROC R package.

### 2.7. Analysis of the Correlation of Tumor-Infiltrating Immune Cells (TIICs) with the BGN Genes

The relationship of TIICs with the BGN genes in GC was investigated by the TIMER dataset (https://cistrome.shinyapps.io/timer/) [23]. Additionally, the relative ratio of different TIICs in each carcinoma sample was calculated by the xCell algorithm [24]. xCell performs cell type enrichment analysis from gene expression data for 64 immune and stromal cell types, which is a gene signature-based method learned from thousands of pure cell types from various sources [24]. The data was presented by R packages “immunedeconv” and “pheatmap.”

## 3. Results

### 3.1. Screening the DEGs in GC

A total of 4397 DEGs in GC samples after comparison with normal samples were identified by analyzing TCGA dataset (Figure 1(a)), with the criteria of *p* < 0.1 and FC > 1.5 (∣log2FC | >0.585). Then, the same cutoff criteria were applied for GEO datasets GSE118897 (Figure 1(b)), GSE19826 (Figure 1(c)), and GSE54129 (Figure 1(d)). And 372, 1313, and 1752 DEGs were identified in GC samples compared to normal samples. The selected DEGs were subjected to the heatmap clustering analysis, and the data are illustrated in Figure 1.

Furthermore, the overlapped DEGs between RNA-Seq profiles and GEO datasets were integrated (Figure 1(e)). We found that 37 genes among these overlapped DEGs were differentially expressed in 4 datasets, including MFSD4A, ERO1B, DNER, CA9, TMED6, CPA2, GUCA2B, GKN1, CAPN13, MAMDC2, ZBTB16, MFAP2, BGN, THY1, THBS2, TIMP1, PRRX1, TMEM158, CLDN1, SALL4, SFRP4, TEAD4, RARRES1, CEMIP, EPHB2, CD300LF, PLPPR4, GREM1, FJX1, CHI3L1, IGF2BP3, WNT2, TREM1, CXCL9, CXCL8, and TREM2 (Figure 1(e)).

### 3.2. PPI Analysis of Differentially Expressed Genes in GC

Then, 36 DEGs were imported into the PPI network complex consisting of 36 nodes and 134 edges in this network (Figure 1(f)). Among them, 17 genes were identified as hub nodes in the network by connecting to more than 2 different genes, including PRRX1, THBS2, MFAP2, BGN, TIMP1, CHI3L1, CXCL9, CXCL8, TREM1, CD300LF, TREM2, and THY1.

### 3.3. The Dysregulation of Hub Genes Was Correlated to Shorter Overall Survival (OS) Time in GC

By analyzing the correlation between OS and gene expression of hub genes using KM methods, we identified that MFAP2, BGN, and TREM1 levels were obviously correlated with OS time in GC. Then, we employed the “survminer” R package to acquire the average cutoff point and classified GC patients into high and low groups.  Figure 2 shows that more dead cases were identified in MFAP2 (Figure 2(a)), BGN (Figure 2(b)), and TREM1 (Figure 2(c)) in highly expressed groups compared to lowly expressed groups (Figures 2(a)–2(c)). The KM survival curves showed that higher levels of MFAP2 (Figure 2(d)), BGN (Figure 2(e)), and TREM1 (Figure 2(f)) exhibited a remarkable correlation with shorter OS time in GC. Next, we applied 1-, 3-, and 5-year receiver operating characteristic (ROC) curve analyses via comparing individual AUC values. The 1-, 3-, and 5-year AUC values for the MFAP2 were 0.538, 0.652, and 0.781 (Figure 2(g)). The 1-, 3-, and 5-year AUC values for the BGN were 0.536, 0.614, and 0.761 (Figure 2(h)). The 1-, 3-, and 5-year AUC values for the TREM1 were 0.542, 0.569, and 0.54 (Figure 2(i)). Our data indicated that MFAP2, BGN, and TREM1 expression could precisely forecast GC patients' prognosis. Among them, BGN was selected for further analysis due to the fact that it has the highest connection score in the PPI network.

### 3.4. Prognostic Nomogram Establishment and Validation of BGN in GC

To explore the feasibility of utilizing the establishment of the prognostic nomogram as an independent predictor of STAD patients' prognosis, we performed univariate and multivariate Cox regression analyses. Univariate analysis data showed that BGN (*p* = 0.00699), age (*p* = 0.00928), and pTNM stage (*p* = 0.00862) forecasted the worse OS (Figure 3(a)). Additionally, our results revealed that BGN was an independent prognostic index of GC patients in TCGA (Figure 3(b)). Next, we constructed a nomogram to predict the 1-year, 3-year, and 5-year OS rates based on univariate and multivariate analyses of BGN (Figure 3(c)). Moreover, the calibration curve indicated good performance in the estimation of 1-year, 3-year, and 5-year OS of the nomogram compared with the estimation of Kaplan-Meier (Figure 3(d)).

### 3.5. Confirmation of BGN by the KM Plotter

The associations of survival data and BGN expression in 5 different datasets were confirmed by KM plotter analysis. Our results showed that higher expression of BGN was correlated to shorter OS than patients with lower BGN expression by analyzing GSE29272 (Figure 4(a)), GSE62254 (Figure 4(b)), GSE14210 (Figure 4(c)), GSE15459 (Figure 4(d)), and Kaplan-Meier plotter (Figure 4(e)) databases. These results suggested that BGN may act as an oncogene in GC.

### 3.6. BGN Expression Was Largely Correlated with TIICs in GC

Next, the correlations of BGN members and TIICs were assessed and the TIMER database analysis data showed that BGN had a markedly negative correlation with B cells but had positive correlations with CD8^+^ T cells, CD4^+^ T cells, macrophages, neutrophils, and dendritic cells in GC samples (Figures 5(a)–5(f)).

In light of the average BGN mRNA expression value in TCGA database, we separated GC samples into BGN highly expressed and BGN lowly expressed groups. We exploited the xCell algorithm to compute the proportion of different TIICs in BGN highly expressed and lowly expressed GC samples.  Figure 5 presents different levels of immune cell infiltration in the abovementioned two BGN groups. The high level of BGN was tightly related to the infiltrating levels of the activated myeloid dendritic cell, T cell CD4^+^ naïve, T cell CD4^+^ central memory, T cell CD8^+^ naïve, common lymphoid progenitor, common myeloid progenitor, myeloid dendritic cell, endothelial cell, macrophage, M1 macrophage, M2 macrophage, mast cell, monocyte, B cell naive, neutrophil, T cell NK, B cell plasma, T cell gamma delta, T cell CD4^+^ Th1, and T cell CD4^+^ Th2 in GC (Figures 5(g)–5(j)). Moreover, we observed that the microenvironment score and stroma score in GC were raised in the BGN high group (Figure 5(j)). Our results implied that BGN probably played as the regulators of the immune microenvironment in GC.

### 3.7. BGN Was Differentially Expressed and Related to Tumor-Infiltrating Immune Cells across Human Cancers

The above analysis demonstrated that BGN was upregulated in GC; however, its prognostic value across human cancers remained largely unclear. For the pan-carcinoma comparisons, we utilized TCGA to explore BGN expression, and the results showed that BGN was expressed in most cancer types, including BLCA, BRCA, CHOL, COAD, DLBC, ESCA, GBM, HNSC, KIRC, LGG, OV, PAAD, READ, SKCM, STAD, TGCT, and UCS, in comparison with its corresponding tumor tissues (Figures 6(a)–6(d)). However, we found that BGN was suppressed in ACC, CESC, KICH, and THCA samples. Collectively, these findings suggested that BGN was a probable novel biomarker for multiple cancer diagnoses.

Next, we analyzed the association between BGN expression and TIICs across human cancers. Using the TIMER database, we found out that the relationship between BGN expression and TIICs was significantly related to B cells, CD8^+^ T cells, CD4^+^ T cells, macrophages, neutrophils, and dendritic cells in multiple cancer types, such as BLCA, BRCA, COAD, ESCA, HNSC, KICH, LGG, LIHC, LUAD, LUSC, OV, PAAD, PCPG, PRAD, READ, SKCM, and STAD (Figure 7(a)). We detected the correlation of the BGN level with immune infiltration based on the xCell dataset. Of interest, we found that BGN expression was significantly positively related to the microenvironment score, stroma score, endothelial cell, macrophage 1 (M1), macrophage 2 (M2), mast cell, monocyte, and myeloid DCs in overall immune cells in various types of human cancers, including BLCA, BRCA, COAD, ESCA, HNSC, KIRC, LGG, LIHC, LUAD, LUSC, PAAD, PCPG, PRAD, READ, SKCM, STAD, TGCT, and THCA. Meanwhile, we observed that BGN expression was significantly negatively related to B cells in more than 80% of cancer types (Figure 7(b)).

## 4. Discussion

GC is the most commonly diagnosed neoplasm of the digestive tract. Although the diagnosis and treatment strategies of GC have been greatly improved in the past few decades, the morbidity and lethality rates of GC are still rising due to lacking early diagnosis strategies and powerful treatments [1]. Most GC cases are related to *H*. *pylori* [25] and EBV infection [4]. A few GC cases exhibited an association with the *CDH1* [26] or *MMR* gene [27], while GC with sporadic mismatch repair defects has an epigenetic silencing of MLH1 in the context of the CpG island methylator phenotype (CIMP) [28]. In our literature, we found a total of 37 DEGs in GC by analyzing 4 independent datasets, including MFSD4A, ERO1B, DNER, CA9, TMED6, CPA2, GUCA2B, FD, CAPN13, MAMDC2, ZBTB16, MFAP2, BGN, THY1, THBS2, TIMP1, PRRX1, TMEM158, CLDN1, SALL4, SFRP4, TEAD4, RARRES1, CEMIP, EPHB2, CD300LF, PLPPR4, GREM1, FJX1, CHI3L1, IGF2BP3, WNT2, TREM1, CXCL9, CXCL8, and TREM2. Of note, several of them had been implied in human cancers. For example, MFSD4 was identified as a putative tumor suppressor in gastric cancer [29]. THY1 acted as a potential novel diagnostic marker for GC [30]. Upregulation of CLDN1 was related to shorter OS in GC [31]. Three hub genes, BGN, TREM1, and MFAP2, were identified to be hub genes in GC. Among them, BGN was chosen for further analysis. Our research has discovered that the overexpression of BGN was correlated to poorly prognostic status and resulted in the increases in immune infiltrating levels in cytotoxic cells, DCs, macrophages, neutrophils, Th17 cells, Th2 cells, etc., in GC. This study for the first time revealed that BGN was a potential biomarker for GC.

So far, a large number of effective biomarkers for GC diagnosis and prognosis have been identified. For instance, by integrative analysis of the Gene Expression Omnibus (GEO) database and TCGA database, Zhang et al. elaborated that UCA1, HOTTIP, and HMGA1P4 lncRNAs were upregulated in GC tissues and firstly identified that HMGA1P4, a target of miR-301b/miR-508, took part in the process of cell cycle and senescence by modulating CCNA2 in GC. This study suggested that the 3 lncRNAs were candidate contributors to the development of GC, and their potential functions perhaps had an association with GC prognosis. Utilizing TCGA and cross-validation with GEO datasets, Lan et al. [32] identified that 9 genes associated with the tumor microenvironment were largely related to poorly prognostic status in GC patients. Using bioinformatics analysis, Chong et al. revealed that abnormally expressed FN1, TIMP1, and SPP1 displayed a relation to poor OS in GC patients [33]. Previous studies have indicated that inhibited FN1 led to the reduction of GC cell invasion and migration [34, 35]. Some reports indicated that the overexpression of TIMP1 facilitated GC cell proliferation in patients via the NF-*κ*B-dependent mechanism [35]. It was demonstrated that the high expression of SPP1 was closely associated with GC occurrence [36]. The advance of modern bioinformatics and high-throughput sequencing tools provides a variety of effective tools for analyzing the molecular mechanism of carcinomas. Here, our literature tried to identify differentially expressed genes in GC by using a series of public datasets. In total, 37 key genes were identified to be differentially expressed in GC. By applying PPI network analysis, BGN, TREM1, and MFAP2 were identified to be hub genes in GC. Further analysis demonstrated that BGN, TREM1, and MFAP2 were upregulated and their levels exhibited a correlation to shorter OS time in patients with GC.

TREM participated in innate immune and inflammatory responses, and TREM1 signaling is activated upon crosslinking its ligand, leading to the production of TNF*α*, IL-18, and CCL2 through the adaptor DAP12 [37]. It was described that TREM1 promoted tumorigenesis and supported tumor growth in multiple tumor models, such as intestinal, pancreatic, and lung carcinomas [38]. TREM1 is also expressed in gastric mucosa epithelial cells and is upregulated in the gastric mucosa of adult patients with *H*. *pylori* infection [39]. MFAP2 is related to modulating the deposition of proelastin on microfibers to shape elastic fibers [40, 41]. Recently, MFAP2's role in carcinoma has attracted much attention. For instance, Wang et al. [40] claimed that MFAP2 promoted the epithelial-mesenchymal transition by motivating the TGF-*β*/SMAD2/3 signaling pathway in GC cells. Shan et al. [42] presented that MFAP2 might exhibit a pivotal role in GC progression and that it is displayed as an oncogene. Yao et al. reported that upregulated MFAP2 was displayed in GC tissues, and this upregulation had a bearing on GC cell proliferation, migration, and invasion.

The 5-year OS rate of early GC is over 90% [1]. However, most patients with GC are diagnosed at a late stage [1]. Herein, exploring the hidden details may be conducive to developing ideal strategies for GC early diagnostics. Microarray and bioinformatics analyses are largely applied in disease diagnosis and drug screening. For instance, using high-throughput screening methods, Li et al. [43] identified that CASR, CXCL12, and SST were potential prognosis markers for GC treatment. In our research, we reported that BGN was significantly upregulated in GC samples. More dead cases were identified in BGN highly expressed groups compared to lowly expressed groups. The KM survival curves showed that higher levels of BGN had a significant correlation with worse prognosis in GC. Moreover, we utilized TCGA to explore BGN expression in pan-cancers and found that BGN was highly expressed in most cancer types. This study revealed that BGN could be utilized as prospective treatment targets and biomarkers for multiple human cancers, especially for GC.

Despite the fact that several previous studies had revealed the potential roles of BGN in GC, the detailed roles of BGN in GC prognosis and immune response remained to be unclear. The neoplasm microenvironment primarily contains the mixture of neoplasm cells and TIICs, extracellular matrix, blood vessels, and other stromal components. Research studies on the neoplasm microenvironment have indicated the role of TIICs in the treatment response and immunotherapy resistance across diverse carcinoma types. The mechanisms by which TIICs participate in the systemic antitumor response are still being explored. Our research showed that BGN had a markedly negative correlation with B cells but had positive correlations with CD8^+^ T cells, CD4^+^ T cells, macrophages, neutrophils, and dendritic cells in GC samples. Moreover, the pan-cancer analysis also demonstrated that BGN was tightly related to the infiltrating levels of various types of tumor-infiltrating immune cells. This study for the first time revealed that BGN was a potential biomarker for GC tumor immune infiltration.

## 5. Conclusion

In conclusion, a total of 37 differentially expressed genes were identified in GC by analyzing TCGA, GSE118897, GSE19826, and GSE54129. Using the PPI database, we identified 17 hub genes in GC. By analyzing the expression of hub genes and OS, MFAP2, BGN, and TREM1 were related to the prognosis of GC. In addition, our results showed that higher levels of BGN exhibited a significant correlation with shorter OS time in GC. Moreover, we revealed that BGN had a markedly negative correlation with B cells but had positive correlations with CD8^+^ T cells, CD4^+^ T cells, macrophages, neutrophils, and dendritic cells in GC samples. The pan-cancer analysis demonstrated that BGN was differentially expressed and related to tumor-infiltrating immune cells across human cancers. This study for the first time revealed that BGN was a potential biomarker for the prediction of GC prognosis and tumor immune infiltration.

## Figures and Tables

**Figure 1:** Screening the hub DEGs in GC. (a–d) A total of 4397, 372, 1313, and 1752 DEGs were identified in GC samples compared to normal samples by analyzing TCGA (a), GSE118897 (b), GSE19826 (c), and GSE54129 (d) datasets. (e) Venn map analysis identified common DEGs in 4 datasets. (f) PPI analysis identified the interaction among common DEGs.

**Figure 2:** The dysregulation of hub genes was correlated to shorter overall survival (OS) time in GC. (a–c) More dead cases were identified in MFAP2 (a), BGN (b), and TREM1 (c) in highly expressed groups compared to lowly expressed groups. (d–f) The KM survival curves showed that higher levels of MFAP2 (d), BGN (e), and TREM1 (f) exhibited a significant correlation with shorter OS time in GC. (g–i) 1-, 3-, and 5-year ROC curve analyses of MFAP2 (g), BGN (h), and TREM1 (i).

**Figure 3:** Prognostic nomogram establishment and validation of BGN in GC. (a, b) Univariate and multivariate Cox regression analyses of BGN in GC. (c) Nomogram to predict the 1-year, 3-year, and 5-year overall survival of GC cancer patients. (d) Calibration curve for the overall survival nomogram model in the discovery group.

**Figure 4:** Confirmation of BGN by the KM plotter. (a–e) Higher expression of BGN was correlated to shorter OS than patients with lower BGN expression by analyzing GSE29272 (a), GSE62254 (b), GSE14210 (c), GSE15459 (d), and Kaplan-Meier plotter (e) databases.

**Figure 5:** BGN expression was largely correlated with TIICs in GC. (a–f) TIMER database analysis data showed that BGN had a markedly negative correlation with B cells (a) but had positive correlations with CD8^+^ T cells (b), CD4^+^ T cells (c), macrophages (d), neutrophils (e), and dendritic cells (f) in GC samples. (g–j) The xCell algorithm was used to compute the proportion of different TIICs in BGN highly expressed and lowly expressed GC samples.

**Figure 6:** BGN was differentially expressed across human cancers. (a) BGN was differentially expressed in ACC, BLCA, BRCA, CESC, CHOL, COAD, DLBC, and ESCA. (b) BGN was differentially expressed in GBM, HNSC, KICH, KIRC, KIRP, LAML, LGG, and LIHC. (c) BGN was differentially expressed in LUAD, LUSC, MESO, OV, PAAD, PCPG, PRAD, and READ. (d) BGN was differentially expressed in SARC, SKCM, STAD, TGCT, THCA, THYM, UCEC, UCS, and UVM.

**Figure 7:** BGN was related to tumor-infiltrating immune cells across human cancers. (a, b) The correlation between BGN expression and tumor-infiltrating immune cells across human cancers by analyzing the TIMER database (a) and xCell dataset (b).

## Data Availability

The data used during the present study are available from the corresponding author upon reasonable request.
